# Effects of the COVID-19 Pandemic on Stroke Patients

**DOI:** 10.7759/cureus.9995

**Published:** 2020-08-24

**Authors:** Hammad Ghanchi, Ariel Takayanagi, Paras Savla, Omid R Hariri, Emilio C Tayag, Michael Schiraldi, Lucille Jorgensen, Dan E Miulli

**Affiliations:** 1 Neurosurgery, Riverside University Health System Medical Center, Moreno Valley, USA; 2 Neurosurgery, Kaiser Permanente-Orange County, Anaheim, USA; 3 Neurology and Neurosurgery, Desert Regional Medical Center, Palm Springs, USA; 4 Neurosurgery, Desert Regional Medical Center, Palm Springs, USA; 5 Neurosurgery, Redlands Community Hospital, Redlands, USA; 6 Stroke Program Coordinator, Arrowhead Regional Medical Center, Colton, USA; 7 Neurosurgery, Arrowhead Regional Medical Center, Colton, USA

**Keywords:** stroke, diagnostic delay, nihss, covid-19, tpa, coronavirus quarantine, transient ischemic attack, patient delay, stroke guidelines, stroke protocol

## Abstract

Introduction

The severe acute respiratory syndrome coronavirus 2 (SARS2-CoV-2) induced pandemic (COVID-19 pandemic) has affected healthcare in all aspects, including stroke care. We sought to investigate this effect with analysis of our hospital’s stroke treatment protocols as well as stroke volume on state, regional, and national levels.

Methods

This was a retrospective review of prospectively collected data from our stroke registry to assess the impact of the SARS2-CoV-2 induced pandemic on the volume of stroke patients presenting to our facility. Demographics collected included age, sex, race, National Institute of Health Stroke Scale (NIHSS) on admission, discharge modified Rankin Score (mRS), type of stroke (ischemic, hemorrhagic, or transient ischemic attack), time of symptom onset, and time to initial imaging. Data were also stratified by date and comparison was made between the intra-COVID-period (March and April 2020), pre-COVID period (March and April 2019), and peri-COVID period (January and February 2020). To determine stroke trends on a national level, we utilized the Get with the Guidelines (GWTG) stroke database to compare stroke volumes in the pre-COVID, peri-COVID, and intra-COVID periods between our hospital, all California hospitals, and the West and Pacific regions.

Results

There was a significant increase in last known well time (LKWT) to arrival to the emergency department (ED) (LKWT to door) as well as time from arrival to the ED to obtaining a computed tomography (CT) of the head (door to CT) in March 2020 compared to 2019 (p=0.0220 and p=0.0475, respectively). There were significantly fewer transient ischemic attacks (TIAs) in California hospitals as well as in March and April 2020 in comparison to January and February 2020 (p=0.0417). Similarly, there were significantly fewer TIAs in March and April 2019 compared to March and April 2020 (p=0.0360). The decrease in TIAs was also seen at our hospital in both time frame comparisons as well as in West Regional Hospitals in March and April 2020 compared to March and April 2019 (p=0.0111, p=0.0215, and p=0.0414, respectively).

Conclusion

Stroke care has been disrupted by the COVID-19 pandemic worldwide. We identified a delay in LKWT to door as well as time from door to CT in March 2020 compared to March 2019 at our institution. There was a statistically significant decrease in final diagnosis of TIA at our hospital, all California hospitals, and all West Regional hospitals during the March-April 2020 window, suggesting that some patients with minor stroke symptoms may not be presenting to the hospital in the midst of the pandemic. Strategies to minimize delays in care and maximize functional recovery must continue to evolve as new challenges are met during the COVID-19 pandemic.

## Introduction

The coronavirus disease 2019 (COVID-19) pandemic caused by the severe acute respiratory syndrome coronavirus 2 (SARS2-CoV-2) has had detrimental effects on not only our economy, but it has also affected treatment of other serious diseases. Recent studies have been published demonstrating the adverse effects this pandemic has had thus far on the treatment of stroke patients [1-4].

Over the past few decades, great measures have been taken to decrease time from stroke symptom onset to treatment in order to maximize recovery [5]. However, during the COVID-19 pandemic, the public has been discouraged from leaving their homes to minimize risk of infection and slow the spread of the disease. A state of emergency was issued by many state governments early March 2020 which evolved into stay-at-home orders. The orders were first placed in California mid-March 2020 and slowly spread to the other states in the following weeks [6]. At the same time, hospitals across the nation started to prepare for a surge in hospitalizations and began focusing efforts on providing COVID-directed care. Since the pandemic began, delays in presentation and decreases in patients receiving tissue plasminogen activator (tPA) have been reported [2]. We performed a retrospective study using our institutional stroke registry to investigate pre- and intra-hospital delays during the COVID period. We then compared our institutional data to the Get with the Guidelines (GWTG) database to analyze our experience by comparing regional and national trends in stroke volume [7,8].

## Materials and methods

This was a retrospective review of the stroke registry at our institution, a Level 1 primary stroke center as certified by the Joint Commission/American Stroke Association in Colton, California, to assess what impact the SARS2-Cov-2 outbreak had on the number of patients presenting with stroke to our hospital. All patients with a final diagnosis of ischemic stroke, transient ischemic attack (TIA), subarachnoid hemorrhage (SAH), or intraparenchymal hemorrhage (IPH) were reviewed.

Demographics were collected including age, sex, race, National Institute of Health Stroke Scale (NIHSS) on admission, discharge modified Rankin Score (mRS), type of stroke (ischemic, hemorrhagic, or transient ischemic attack), last known well time (LKWT), and time to initial cranial imaging. Data was also stratified by date into three groups: (a) intra-COVID period (March and April 2020), (b) pre-COVID period (March and April 2019), and peri-COVID period (January and February 2020).

To determine stroke trends on a regional and national level, we utilized the GWTG database to compare stroke volumes in the same three time periods between our hospital, all California hospitals, all Pacific hospitals (Alaska, Washington, Oregon, California, and Hawaii), all Western hospitals (Pacific plus Montana, Idaho, Wyoming, Nevada, Utah, Colorado, Arizona, and New Mexico), and all hospitals in the United States that submit data to the registry. The numbers of patients presenting to these hospitals with a final diagnosis of ischemic stroke, TIA, SAH, or IPH were reviewed.

The primary endpoint of this study is to compare whether there was a significant change in the number of patients presenting to our institution with stroke during the SARS2-CoV-2 pandemic. The secondary endpoints were to assess differences in severity of stroke, delays in imaging, delays in presentation, and changes in stroke incidence.

Statistical analysis was performed using Student’s t-Test to compare the sample means and assess for any significant differences in the patient volumes, times for treatment, and severity of strokes.

## Results

County Hospital Stroke Results

On our review, 348 patients presented to our institution between during the first four months in 2019 and 302 patients in 2020 with symptoms concerning for stroke resulting in activation of our stroke protocols. Of these patients, a total of 262 were found to have a final diagnosis of stroke (ischemic, hemorrhagic, or TIA) on discharge; 135 patients in 2019 and 127 patients in 2020. The mean age of both groups was 60 years with 2019 ranging from 20 to 99 years old and 2020 ranging from 21 to 93 years old. For gender, no significant differences were seen, with 2019 having 67 (49.6%) males and 68 (50.4%) females and 2020 having 57 (44.9%) males and 70 (55.1%) females.

There was a significant increase in last known well time (LKWT) to arrival to the emergency department (ED) (LKWT to door) as well as time from arrival to the ED to obtaining a computed tomography (CT) of the head (door to CT) in March 2020 compared to 2019 (p=0.0220 and p=0.0475, respectively) (Table 1, Figure 1, Figure 2). There was no difference in LKWT to door or door to CT between April 2019 and 2020. Additionally, while the NIH score was increased in April 2020 compared to 2019 from 4.14 to 8.16, the difference was not statistically significant (p=0.17) (Table 1, Figure 3).

**Table 1:** Comparison of pre-COVID versus COVID period timing and stroke severity Abbreviations: LKWT: last known well time, NIH: National Institutes of Health, H&H: Hunt and Hess score, ICH: Intraparenchymal hemorrhage score, mRS: modified Rankin scale, Pre-COVID: March, April 2019, COVID period: March, April 2020, N/A: not applicable

Month	Mar '19	Mar '20			Apr '19	Apr '20	
	Mean	Mean	p-value		Mean	Mean	p=value
Timing							
LKWT to door (min)	836	2561	0.0220		1457	1039	0.4623
Door to CT (min)	17	76	0.0475		50	57	0.8321
Admission Stroke Severity and Discharge Functional Status							
NIH	6.27	5.74	0.8173		4.14	8.16	0.1767
mRS	2.08	2.43	0.4900		2.32	2.32	0.9882

**Figure 1:** Last Known Well Time to Door

**Figure 2:** Time from Door to CT

**Figure 3:** Stroke Severity and Functional Status

National, Regional, and Local Stroke Volume

Stroke volumes in January through April of 2019 and 2020 for our hospital as well as regional and national data are listed in Table 2. Comparisons of stroke volumes in the peri-COVID period and the COVID period as well as pre-COVID period and COVID-period are demonstrated in Table 3. There were significantly fewer TIAs in California hospitals as well as in March and April 2020 in comparison to January and February 2020 (p=0.0417). Similarly, there were significantly fewer TIAs in March and April 2019 compared to March and April 2020 (p=0.0360). The decrease in TIAs was also seen at our hospital in both time frame comparisons (p=0.0111, p=0.0215) as well as in West Regional Hospitals when March and April 2020 was compared to March and April 2019 (p=0.0414). There was also a significant decrease in ischemic strokes in the Pacific region from March/April 2019 to March/April 2020 and from January/February 2020 to March/April 2020 (p=0.0462 and p=0.0383, respectively).

**Table 2:** National, regional, and local stroke volumes in 2019 and 2020 Abbreviations: ARMC: Arrowhead Regional Medical Center; IS: ischemic stroke; TIA: transient ischemic attack <24 hours; SAH: subarachnoid hemorrhage; ICH: intraparenchymal hemorrhage; All hospitals: all hospitals in the US; Pacific: Alaska, Washington, Oregon, California, Hawaii; West Region: Pacific region plus Montana, Idaho, Wyoming, Nevada, Utah, Colorado, Arizona, New Mexico

		IS			TIA			SAH			ICH	
Region		2019	2020		2019	2020		2019	2020		2019	2020
ARMC												
January		14	14		13	15		3	0		3	9
February		21	15		8	16		1	2		7	10
March		11	11		12	6		1	4		11	9
April		12	14		13	4		0	1		5	5
CA Hospitals												
January		4086	4325		658	700		277	270		909	912
February		3705	3881		641	659		271	238		868	785
March		4115	3475		717	458		275	202		866	747
April		3987	2284		680	349		257	160		825	508
Pacific Region												
January		5821	6037		945	940		387	360		1233	1211
February		5176	5408		929	894		363	304		1164	1083
March		5831	4941		1036	600		366	284		1135	997
April		5636	3263		951	426		361	218		1087	716
West Regional												
January		7901	8172		1249	1189		540	492		1611	1623
February		6982	7372		1194	1126		494	422		1511	1447
March		7824	6634		1344	764		496	380		1505	1329
April		7599	4474		1222	525		501	280		1459	951
All Hospitals												
January		40644	42660		6749	7150		2383	2353		7305	7287
February		36946	37999		6194	6556		2135	1940		6489	6233
March		40403	34986		7340	4940		2269	1960		6890	5819
April		40099	22748		6877	2856		2174	1431		6538	4307

**Table 3:** Comparision of national, regional, and local stroke volumes in pre-COVID, peri-COVID, and COVID periods (p values) Abbreviations: ARMC: Arrowhead Regional Medical Center; IS: ischemic stroke; TIA: transient ischemic attack <24 hours; SAH: subarachnoid hemorrhage; ICH: intraparenchymal hemorrhage; All hospitals: all hospitals in the US; Pacific: Alaska, Washington, Oregon, California, Hawaii; West Region: Pacific region plus Montana, Idaho, Wyoming, Nevada, Utah, Colorado, Arizona, New Mexico

	IS	TIA	SAH	ICH
ARMC				
Jan Feb '20 vs Mar Apr '20	0.3333	0.0111	0.4929	0.3491
Mar Apr '19 vs Mar Apr '20	0.5918	0.0215	0.3333	0.8075
California Hospitals				
Jan Feb '20 vs Mar Apr '20	0.1941	0.0417	0.1097	0.2440
Mar Apr '19 vs Mar Apr '20	0.1896	0.0360	0.0653	0.2140
Pacific Region				
Jan Feb '20 vs Mar Apr '20	0.0462	0.2022	0.1729	0.1986
Mar Apr '19 vs Mar Apr '20	0.0383	0.0767	0.0781	0.2143
West Regional				
Jan Feb '20 vs Mar Apr '20	0.1940	0.0534	0.1729	0.1986
Mar Apr '19 vs Mar Apr '20	0.1853	0.0414	0.0781	0.2143
All Hospitals				
Jan Feb '20 vs Mar Apr '20	0.2221	0.1123	0.3111	0.2069
Mar Apr '19 vs Mar Apr '20	0.2040	0.0950	0.1894	0.1673

## Discussion

SARS2-CoV-2 is the first virus in modern history to cause a global economic shutdown. In addition to its effect on the economy, SARS2-CoV-2 also caused major disruptions in healthcare as many hospitals were forced to cancel elective surgeries and postpone outpatient and specialty appointments to conserve personal protective equipment (PPE) and reduce exposure risk. Teo et al. has suggested that the recent change in healthcare has had a significant impact on care of stroke patients [2].

A delay in management of stroke patients may be related to the COVID-19 pandemic. Schirmer et al. compared stroke severity and time to presentation between patients who presented with stroke in the pre-COVID and intra-COVID period at twelve institutions, and the corresponding months from one year prior [9]. There was a significant increase in time interval between symptom onset and time to presentation to a stroke center. Patients in the baseline period presented in 442 minutes (mins), while intra-COVID period patients presented in 603 mins. In the present study, the LKWT to ED door significantly increased in March 2020 compared to March 2019 (2561 mins versus 836 mins, p=0.0220); this corresponds to when the State of Emergency was declared and most states issued stay-at-home orders.

Another study showed similar results with a significant increase in LKWT to door time during the COVID-19 period, and more importantly a significant reduction in patients who arrived within the 4.5 hour tPA window [2]. Similarly, Kerleroux et al. also found that patients who were treated during the same time period were less likely to receive tPA [3]. While the cause of delay in presentation is unclear, it may be related to reluctance to go to the hospital due to fear of infection [2]. Another possibility is that there is a delay in ambulance response times, but further studies will be necessary to identify the cause of the delays. Mechanical thrombectomy times have also been adversely affected. Kerleroux et al. showed a significant decrease in thrombectomy volumes as well as a significant increase in time between imaging and groin puncture <0.001) [3]. The authors hypothesize that the decrease in number of thrombectomies may be related to the saturation of transport systems, which may prevent patients from being transferred to facilities capable of stroke thrombectomies in a timely manner [3]. Institutional delays during the pandemic, as seen in our study, may result in further delays.

We also found a statistically significant increase in time from door to CT when March 2019 and March 2020 were compared (17 mins to 76 mins, p=0.0475). When patients who are suspected of having SARS2-CoV-2 infection undergo a CT study at our hospital, the CT scanner room must undergo strict disinfecting protocols before another patient can be scanned. This may have caused delays in CT scans overall. Interestingly, there was no significant difference in time from door to CT between April 2019 and April 2020 (p=0.8321). This corresponds with the development and distribution of the rapid COVID-19 test during April which may have helped to minimize CT downtime. Furthermore, our times for April 2019 were higher than average, which may account for the decrease being smaller than the decrease from March 2019 to March 2020. Turin et al. have also shown in the past that incidence of stroke in the spring season is higher [10]. Another delay that may be related to the pandemic is the additional time needed for donning and doffing of personal protective gear. However, these explanations are anecdotal and future studies are necessary to elucidate the causes of in-hospital delays.

There was no significant difference in LKWT to door time when April of 2020 was compared to April 2019 (p=0.4623). However, we do see a decrease in number of patients diagnosed with stroke during this month, trending down from March in almost all regions (Table 2). Moreover, there was a statistically significant decrease in final diagnosis of TIA at our hospital, all California hospitals, and all West Regional hospitals during the March-April 2020 window (Table 3). Those with minor or transient stroke-like symptoms (i.e. TIAs) may have avoided presenting to the hospital due to fear of infection. With regards to severity of stroke, we found that NIHSS scores were higher in April 2020 (8.16) than April 2019 (4.14), but the difference did not reach statistical significance (p=0.1767). There was also no significant difference in NIHSS score between March 2019 and March 2020 (p=0.8173). This was consistent with Schirmer et al. who reported no change in NIH score from 2019 [9]. Finally, the patient outcomes as measured by mRS were similar between March and April 2019 and March and April of 2020 (p=0.49) (Table 1). 

The AHA/ASA Stroke Council Leadership has published guidelines for care of stroke patients during the COVID-19 pandemic. While the recommendation is to continue to follow stroke protocols and aim to minimize time to treatment, they suggest that the guidelines should be treated as goals rather than expectations given limited resources and staffing [11]. Other efforts have been made to streamline stroke care during the pandemic. Khosravani et al. published a “Protected Code Stroke” algorithm for managing patients with suspected COVID-19 infection [12]. The authors recommend infectious screening in the field prior to arrival, appropriate use of personal protective equipment, and strategies to minimize exposure during airway management such as early intubation [12]. The Neuroscience in Anesthesiology and Critical Care and Society of Neurointerventional Surgery have recommended rapid COVID-19 testing prior to most neurointerventional procedures. However, given that stroke thrombectomies must be done emergently due to the time-sensitive nature of cerebral ischemia, patients should be assumed to be COVID-19 positive and only essential personnel should be present in the angiography suite [13]. Others have recommended consolidating imaging studies to minimize staff exposure [14]. 

## Conclusions

Stroke care has been disrupted by the COVID-19 pandemic worldwide. We identified a delay in LKWT to door as well as time from door to CT in March 2020 compared to March 2019 at our institution. There was a statistically significant decrease in final diagnosis of TIA at our hospital, all California hospitals, and all West Regional hospitals during the March-April 2020 window, suggesting that some patients with minor stroke symptoms may not be presenting to the hospital in the midst of the pandemic. Strategies to minimize delays in care and maximize functional recovery must continue to evolve as new challenges are met during the COVID-19 pandemic.
